# Cervical Spondylopathy and Lumbar Intervertebral Disc Herniation Coexist in Free Radical Metabolism and Focus Separation in the Body

**DOI:** 10.1155/2021/1480282

**Published:** 2021-11-27

**Authors:** Song Yan, Tian Taotao, Yun Shunwei, Li Haitao, Chang Cheng

**Affiliations:** ^1^Urumqi Friendship Hospital, Xinjiang 830049, China; ^2^Luoyang Orthopedic-Traumatological Hospital of Henan Province (Henan Provincial Orthopedic Hospital), Luoyang 471002, China

## Abstract

Lumbar disc herniation is a common lumbar disease in clinics, which is related to improper use of lumbar vertebrae and osteoporosis. Surgical removal of nucleus pulposus and maintenance of lumbar structural stability are important for the treatment of lumbar disc herniation. At present, in clinical percutaneous intervertebral foramen endoscopic surgery for lumbar disc herniation, interlaminar and intervertebral foramen approaches can be selected. Different approaches have different degrees of difficulty in the treatment of lumbar disc herniation, and the clinical effects that may be obtained are different. In this study, we observed the influencing factors of plasma nitric oxide (NO) and free radical metabolism in patients with lumbar disc herniation and the correlation between the effects of focus separation. The organic combination of local and total illness differentiation and dialectics, conventional acupuncture, and electrical stimulation was highlighted in this study, which linked local acupoints squeezed by nerve roots with distant acupoints along meridians. The use of authoritative quantitative standards and a multifactor assessment of the disease can accurately represent the disease's severity. The patient's condition changes in each period may be expressed more accurately, thoroughly, and objectively through the rise or reduction of the score, making self-evaluation easier for the patient. Electroacupuncture at point may be one of the most important strategies to minimize free radical damage, based on changes in plasma levels.

## 1. Introduction

Lumbar disc herniation refers to a group of syndrome mainly caused by lumbar disc annulus rupture, protruding into the spinal canal, pressing the dural sac or spinal meridian root, causing low back pain, femoral nerve, or sciatica [1]. It is a common clinical disease with a high recurrence rate, which seriously affects the work and life of patients. In the treatment of lumbar disc herniation, nonoperative treatment occupies the primary position, in which acupuncture has achieved a positive effect in the treatment of lumbar disc herniation. The main pathophysiological changes are intervertebral disc degeneration caused by long-term acute and chronic injury, and in the process of its occurrence and development there is an obvious disturbance of microcirculation and local blood flow slows down or even stagnates [2]. The lumbar vertebrae have a large range of motions, which is a stressed part. Severe intervertebral disc wear is easy to cause ischemia, hypoxia, and acute and chronic aseptic inflammation, while the pressure of the intervertebral disc is reduced and the blood supply can be improved when lying down. Therefore, repeated ischemia-reperfusion can be caused locally. During acute and chronic inflammation and ischemia-reperfusion injury, the production of free radicals and lipid peroxidation is increased, resulting in chronic injury of tissues and cells [3].

Long-term free radical injury may be the cause of intervertebral disc degeneration and hyperosteogeny. Some studies have shown that NO is involved in the occurrence and development of pathological and physiological processes [4]. NO has the dual functions of cellular biological messenger molecules and cytotoxic factors; on the other hand, NO has the characteristics of free radicals and can react with oxygen free radicals to form a series of free radicals and nitro compounds with important physiological and pathological functions [5]. Oxygen free radicals can attack polyunsaturated fatty acids in biofilms and trigger lipid peroxidation, resulting in the formation of lipid peroxides [6]. Lipid peroxidation not only transforms reactive oxygen species into active molecules, such as nonfree radical lipid breakdown products, but also enhances their impact through chain or chain branching chain processes [7]. Therefore, the initial reactive oxygen species can lead to the formation of many lipid decomposition products, some of which can cause cell metabolism and dysfunction or even death [8]. Oxygen free radicals may harm cells not only by peroxiding polyunsaturated fatty acids in the biofilm, but also by releasing lipid hydroperoxide breakdown products. It plays a crucial function in the oxidation-antioxidation balance. This enzyme can catalyze the conversion of superoxide free radicals into oxygen and hydrogen peroxide, scavenge superoxide anion radicals, and protect cells from immune injury [9]. The content is an important indicator of the ability of peripheral nerve tissue of resisting the influence of free radicals. The activity is closely related to inflammation and autoimmune diseases. Testing the level of MDA can often reflect the degree of lipid peroxidation in tissue and indirectly reflect the degree of cell injury. The determination often cooperates with that [10]. The activity indirectly reflects the ability of the body of scavenging oxygen free radicals, while the level indirectly reflects the severity of cell attack by free radicals. Electroacupuncture may not only lower NO levels but also enhance activity, according to the findings. On the one hand, it can directly eliminate too many free radicals; on the other hand, it can restore the metabolism of free radicals to normal and effectively prevent the damage of free radicals to the intervertebral disc [11]. By improving the disturbance of microcirculation and the state of hemorheology, we can reduce the pressure in the intervertebral disc, directly improve the clinical symptoms, and block the vicious circle of ischemia-reperfusion injury and free radical damage-microcirculation disturbance, free radical damage in the pathological process. The most frequent illness in clinic is lumbar disc herniation (LIDP), which has the greatest prevalence in spinal orthopaedics, and its detection may be referred to as in Figure 1. In recent years, with the influence of work and life style, it shows an increasing trend year by year. Young and middle-aged manual workers have a high incidence of lumbar disc herniation, whose main clinical manifestations are lumbar and leg pain, scoliosis, dyskinesia, lower limb pain, and numbness, often occurring repeatedly, bringing a heavy burden to patients [12]. The main cause of lumbar disc herniation is intervertebral disc degeneration caused by changes in the microstructure of intervertebral disc tissue, nucleus pulposus herniation, and then compression or stimulation to related nerves, resulting in a series of pains and dysfunctions, seriously affecting the quality of life of patients [13]. The study found that there was no significant difference in the long-term effect of surgical and nonoperative treatment in patients with lumbar disc herniation. At present, it is recognized that the main treatment of lumbar disc herniation is nonoperative treatment [14]. On the other hand, proteomics studies the characteristics of proteins from a macroperspective, including protein mediation, response, function, composition, translation, and interaction between proteins [15–18]. This offers information on the incidence, progression, and molecular metabolism of illnesses at the protein level, which may help us comprehend the information of proteins in a certain condition and investigate the connection between proteins and disease occurrence and progression [19].

Therefore, in order to find the comprehensive pathophysiological mechanism of lumbar disc herniation, it is necessary to identify the differentially expressed proteins [20]. Proteomics technology has developed rapidly in recent years, and there has been an opportunity to synchronously screen differentially expressed proteins associated with disease occurrence, diagnosis, and treatment and posttreatment assessment. This technique is based on a high-throughput, high-performance liquid chromatography-tandem mass spectrometry (HPLC-MS) approach that can detect the relative or absolute concentration of proteins in up to 8 distinct samples at the same time and has a high protein detection rate [21]. It is especially suitable for the study of low-abundance proteins that determine treatment-related differences. Therefore, the study of proteomics technology in the field of treatment of lumbar disc herniation can provide new ideas for the study of the mechanism of treatment of lumbar disc herniation [22]. This study is based on proteomics to carry out the study of nonoperative treatment of lumbar disc herniation with integrated traditional and western medicine, in order to find the difference of protein expression both before and after treatment and then provide a molecular basis for elucidating the related mechanism of integrated traditional and western medicine treatment of the disease. Lumbar disc herniation is a common lumbar disease in clinic, which is related to improper use of lumbar vertebrae and osteoporosis. Surgical removal of nucleus pulposus and maintenance of lumbar structural stability are important for the treatment of lumbar disc herniation. At present, in clinical percutaneous intervertebral foramen endoscopic surgery for lumbar disc herniation, interlaminar and intervertebral foramen approaches can be selected. Different approaches have different degrees of difficulty in the treatment of lumbar disc herniation, and the clinical effects that may be obtained are different. Apolipoprotein A-IV, apolipoprotein B, and apolipoprotein Amuri are the proteins involved in this pathway, with apolipoprotein B being the most highly expressed and apolipoprotein A-IV and apolipoprotein Amuri being the least. When these proteins are enriched in the signal pathways of fat digestion and vitamin digestion and absorption, vitamin metabolic pathways are not involved, which suggests that these three lipoproteins mainly mediate the related effects through fat digestion and absorption pathways. Studies have shown that inhibiting the expression of inflammatory factors by regulating lipid metabolism can improve the symptoms of patients with lumbar disc herniation.

## 2. Analysis of Free Radical Metabolism and Signal Pathway

### 2.1. Complement and Coagulation Cascade

The proteins involved in this pathway are complement core protein-3 (C3), complement C4A, bromine domain protein 4, DNA protein, human *α*-1 antitrypsin protein, and mannose-binding protein C. Among them, bromine domain protein 4, human *α*-1 antitrypsin protein, and mannose-binding protein C are low expressed, while complement C3, complement C4A, and DNA proteins are highly expressed. The complement-coagulation cascade pathway enriched by these proteins mainly contains complement system, coagulation system, and kallikrein kinin system which can be compared with the CT mapping as shown in Figure 2. After searching the database, there is no clear evidence showing the correlation between the coagulation system and kallikrein kinin system and the treatment of lumbar disc herniation, as discussed in the complement system proteins above. Many researchers have shown that the complement system has a role in the treatment of lumbar disc herniation, particularly complement C3, which has been linked to the physiological and pathological processes of lumbar disc herniation. On the other hand, as shown in the protein network diagram, complement C3 is widely related to other proteins and plays a key role in molecular expression. Therefore, it is suggested that complement C3 may be a potential molecular target for nonoperative therapy of integrated traditional and western medicine in the treatment of lumbar disc herniation.

Apolipoprotein C-III, apolipoprotein A-II, and apolipoprotein Amuri are the proteins implicated in this pathway, with apolipoprotein Amuri being downregulated and apolipoprotein C-III and apolipoprotein A-II being upregulated. PPAR-/RXR, PPAR-/RXR, and PPAR-/RXR are the three signal pathways enriched by these proteins, whereas apolipoprotein Amuri III, apolipoprotein Amuri II, and apolipoprotein Amuri are exclusively engaged in the metabolism of the PPAR-/RXR pathway as lipid transport target genes. After searching the database, there is no clear evidence of a link between the PPAR-/RXR pathway and the treatment of lumbar disc herniation, implying that whether these three lipoproteins mediate the related process of lumbar disc herniation via the PPAR-/RXR pathway needs to be investigated further. Apolipoprotein A-IV, apolipoprotein B, and apolipoprotein Amuri are the proteins involved in this pathway, with apolipoprotein B being the most highly expressed and apolipoprotein A-IV and apolipoprotein Amuri being the least. Vitamin metabolic pathways are not involved in the signal pathways of fat digestion and vitamin digestion and absorption in which these proteins are enriched, which suggests that these three lipoproteins are mainly mediated by fat digestion and absorption pathways. Studies have shown that inhibiting the expression of inflammatory factors by regulating lipid metabolism can improve the symptoms of patients with lumbar disc herniation as shown in Figure 3.

By studying the relationship between intervertebral disc degeneration and lipid metabolism in rats, we found that the level of lipid metabolism can regulate the degeneration of intervertebral disc nucleus pulposus. Wang Hong compared the triglyceride levels in the biochemical indexes of patients with lumbar disc herniation to those of healthy individuals and discovered that the triglyceride levels in the biochemical indexes of patients with lumbar disc herniation were greater than those of normal subjects. Deficiency in lipid metabolism occurred in patients with lumbar disc herniation. Apolipoprotein A-IV, apolipoprotein B, and apolipoprotein Amuri, on the other hand, play a critical role in molecular expression, as seen in the protein network diagram. It is suggested that apolipoprotein A-IV, apolipoprotein B, and apolipoprotein Amuri may regulate the nonoperative therapy of integrated traditional and western medicine in the treatment of lumbar disc herniation through fat metabolism, and they may become potential molecular markers in the treatment of lumbar disc herniation.

### 2.2. Receptor Action Signal Pathway

In this experiment, the protein involved in this pathway is fibronectin 1, which is upregulated. Fibronectin 1 is involved in receptor signal pathways such as protein, granulocyte protein, proteoglycan, cell adhesion, and binding. Syndecan is one of the target proteins, which belongs to the heparan sulfate transmembrane proteoglycan family, and Syndecan-4 is an important member of the family. Syndecan-4 can decrease the formation of extracellular matrix and impair the differentiation and regeneration of articular cartilage in the process of articular cartilage degeneration. The nucleus pulposus cells of intervertebral disc are also a kind of highly similar cells of chondrocytes, which are relatively consistent with articular cartilage in gene expression and function. Echtermeyer et al. found that Syndecan-4 promotes the degradation of proteoglycans by upregulating the activity of ADAMTS-5, which leads to cartilage degeneration.

Some researchers have recently looked into the relationship between Syndecan-4 expression in the nucleus pulposus of lumbar intervertebral disc degeneration and the pathological process of lumbar intervertebral disc degeneration. By suppressing the expression of Syndecan-4, it can postpone the degeneration of the nucleus pulposus of the intervertebral disc. Fibronectin 1, on the other hand, is intimately linked to other proteins and plays a vital role in molecular expression, as seen in the protein network diagram. It is proposed that fibronectin 1 may play a role in the production of ECM target protein through the Syndecan receptor signal pathway in the treatment of lumbar disc herniation and that fibronectin 1 may become a serum molecular marker in the treatment of lumbar disc herniation. In this study, the application of nonoperative combination of traditional and western medicine in the treatment of LIDP is effective and worthy of clinical application. In this study, labeling combined with technique was used to screen 21 proteins that were significantly differentially expressed in LIDP before and after nonoperative treatment with integrated traditional and western medicine. Bioinformatics analysis showed that 25 signal/metabolic pathways related to 14 differential proteins were enriched. After verification of related literature reports and comprehensive analysis of bioinformatics, it is suggested that complement C3, fibronectin 1, apolipoprotein A-IV, apolipoprotein B, and apolipoprotein Amuri are likely to be serum markers of combination of traditional and western medicine in the treatment of lumbar disc herniation [23, 24].

## 3. Key Differential Proteins of the Cervical Vertebrae and Lumbar Vertebrae

### 3.1. Bromine Domain Protein

Bromine domain protein 4 is a functional protein that can specifically recognize acetylated lysine in the BET protein group. Recent reports have also pointed out that BET protein also has potential research value in inflammation and autoimmune diseases. As mentioned earlier, it can specifically induce chromatin modification proteins and mediate the activation of related factors, resulting in processes based on expression, transcription, and cell program cycle as shown in Figure 4. A variety of different functional regions that make up it can specifically recognize many transcriptional regulatory factors, which play a role in cell growth and reproduction, chromatin synthesis and assembly, inflammatory response, and oxidative stress. Among them, the bromine domain (BD) can promote the expression of IL-2 and IL-8 and increase their transcriptional activity, thus regulating the inflammatory response. Through the research of inflammatory activation of vascular endothelial cells and its associated mechanism, we discovered that BET protein plays a role in transcriptional control of inflammatory genes by modulating the transcriptional activity of signal pathway. By cultivating human esophageal cancer cells in vitro and targeting the biological activity with a small molecule inhibitor, Wu Dan can limit the proliferation of esophageal cancer cells, therefore downregulating endogenous BRD's biological activity. It demonstrates that BRD4 might be a target for molecular therapy. Despite the fact that numerous studies have demonstrated that BRD4 can be utilized as a therapeutic target for malignant tumors and fibrosis, it has not been linked to lumbar disc herniation in recent years. BRD4 protein expression was shown to be substantially lower before and after nonoperative treatment of lumbar disc herniation using a combination of traditional and western medicine. It is suggested that BRD4 protein may be involved in the process of nonoperative treatment of lumbar disc herniation with integrated traditional and western medicine, but the reason and mechanism of its downregulated expression before and after treatment need to be further studied.

### 3.2. Complement System Protein

Complement system is composed of more than 30 kinds of soluble proteins, membrane-bound proteins, and complement receptors, which mainly participate in the immune response mechanism of the body. Complement system is an indispensable part of human innate immunity and a host defense system with cytotoxic effect, which plays an important role in inflammatory response. Its overactivation can aggravate inflammatory response and cause tissue damage. The bypass, classical, and mannose-binding lectin pathways may all activate the complement system. Human serum contains the main component complement, C3. It functions as a molecular node in the complement activation pathway and may trigger an atopic immune response while also engaging in a nonspecific immunological response. Complement C3, as a key mediator in the complement system, has many binding sites with other molecules and is an important inflammatory transmitter. The main activation products of complement C3 activation cascade include C3a and C4a, which can bind to the corresponding receptors on the surface of mast cells, basophils, and smooth muscle cells, cause cell degranulation, and dilate blood vessels and contract smooth muscle. Its activation product C3a may cause leukocyte infiltration and activation, as well as an increase in the synthesis and release of oxygen free radicals and lysosomal enzymes, which leads to the production of inflammatory factors including tumor necrosis factor and interleukin, which causes tissue edema. Complement C4 is an important component of classical pathway activation, and C4a, as a cleavage product of complement C4, also has the ability of allergic toxin. Studies have shown that C4a has dissolving, scavenging, and immunomodulatory functions of immune complex. DNA protein is a high similarity protein of human complement factor. CFH protein is a complement regulatory molecule that plays a key role in complement activation cluster. This protein is mainly produced in human liver, fibroblasts, and platelets. It can play a role in complement regulatory activity in the complement bypass activation pathway in the first immune response and can play a key role in determining complement C3b activation response by regulating the activation and production of C3 invertase in vivo. On the other hand, as a cofactor, it can increase the degradation of C3b and lose its activation in the cleavage process of C3b. It plays a key role in the early immune response of infectious and autoimmune diseases. The study shows that complement factor H not only participates in inflammation but also regulates glucose and lipid metabolism by activating the para-complement pathway and changing its pathway components. Mannose-binding lectin, also known as mannose-binding protein, is a serum glycoprotein mainly produced by hepatocytes, which is composed of several identical polypeptide chains. It can mediate MBL key recognition of corresponding receptors through terminal-specific binding regions and further induce the activation of a new pathway-lectin pathway, which is different from classical pathway and bypass pathway. It is an important component of nonspecific immune response. In the process of complement activation by MBL pathway, serine protease-2 is directly activated without the participation of antigen and antibody. The activated serine protease-2 can effectively cleave C4 and C2 to produce C3 lyase, thus activating complement cascade enzyme reaction. In the complement activation procedure, MBL is mainly activated by contact with mannose and other corresponding receptors on the surface of pathogenic microorganisms and then cleaves the complement successively according to the cascade enzymatic reaction to form a membrane attack complex. Some studies have detected the level of MBL pathway complement activation product-membrane attack complex in the urine of diabetic patients and found that membrane attack complex sublytic type can activate a series of signal transduction processes and upregulate the expression of various inflammatory factors. Some scholars have reported that the downregulation in deficient mice can inhibit the expression of inflammatory transmitters such as tumor necrosis factor-*α* and interleukin-6, resulting in insensitive inflammatory response caused by certain bacteria and more likely to be infected. MBL's C-terminal sugar recognition domain was previously thought to be used primarily to identify pathogenic microorganisms and their apoptotic cells and to regulate phagocytosis through interactions with immune cells, and that the C-terminal recognition domain would never bind to healthy cells. The comparison results between observation and experiment results can be seen in Figure 5. Recent evidence shows that it can rely on its C-type lectin site to bind to B lymphocytes and dendritic cells by Ca^2+^ attachment mode and regulate the maturation of dendritic cells by regulating nuclear transcription factor signal pathway.

As can be seen, MBL possesses immunological control, complement activation, and inflammatory response regulatory activities. MBL's serum upregulation activity is linked to inflammatory disorders, and overactivation can cause tissue damage. However, there is no definitive proof that it is linked to lumbar disc herniation, and we discovered that mannose-binding protein C is linked to the etiology and pathological process of ankylosing spondylitis. Other research studies have now demonstrated that the complement pathway is linked to the inflammatory response of rheumatoid arthritis and that its serum level has a certain reference importance for rheumatoid arthritis early diagnosis. As a result, this study discovered that complement C3, complement C4a, DNA protein (human complement factor H high similarity protein), and mannose-binding protein C were significantly different before and after combined traditional and western medicine and nonoperative treatment of lumbar disc herniation and that complement C4a, complement factor H, and mannose-binding protein C all played a role in inflammation, immune regulation, and other diseases. However, no conclusive evidence linking it to lumbar disc herniation has been discovered. Complement C3, being a key activating protein of the complement pathway, not only serves as a molecular switch in the complement cascade reaction but also serves as an inflammatory transmitter. Many researchers think it is significant in the etiology, pathological process, and symptoms of lumbar disc herniation in recent years.

### 3.3. Human *α*-1 Antitrypsin Protein

*α*-1-Antitrypsin is a single-chain glycoprotein synthesized by the liver and an important serine protease inhibitor in human plasma. Its main function is to antagonize the activity of proteolytic enzyme so as to prevent normal tissue from being degraded and destroyed by it. Human *α*-1 antitrypsin (HAAT) factor is encoded by Serpin A1 gene; that is to say, the epigenetic fragment of HAAT screened in this study is Serpin A1. Recently, according to several studies, AAT may suppress the production of cytokines, complement activation, and immune cell infiltration in addition to downregulating the expression of different enzymes in serum such as elastase, trypsin, plasma, and thrombin. AAT is a protein that inhibits serine proteases and plays an essential function in the body. It may not only antagonize inflammatory response by antagonising neutrophil elastase, but can also directly act on inflammatory cells such as monocytes and dendritic cells to suppress inflammatory reaction because it possesses vascular permeability activity. At the same time, as an acute phase protein, AAT also has independent anti-inflammatory ability, can block the proinflammatory response of phagocytic neutral peptide, and can regulate the expression of proinflammatory cytokines such as tumor necrosis factor-*α*, interleukin-6, and interleukin-8. When the body has inflammation, infection, cachexia, and other conditions, the blood concentration of AAT will increase by 3 to 4 times, which is often used as a marker of inflammatory reaction. On the other hand, pain is the main clinical manifestation of LIDP patients. Some studies have found that inflammation plays an important role in neurobehavioral changes such as LIDP numbness and root pain. In recent years, through further discussion on the related mechanism of AAT, some scholars have shown that AAT is a multifunctional protein with potential therapeutic function for many kinds of diseases; for example, AAT can play a significant role in the treatment of autoimmune diseases such as rheumatoid arthritis by regulating immune function and inflammatory response. At the same time, the combined application of AAT and doxycycline can also have a considerable effect on arthritis. AAT mediates downregulation of caspase-3 response, thus resisting islet *ß*-cell apoptosis and playing a therapeutic role in type 1 diabetes. AAT may also inhibit the production of caspase-3 and caspase-8 in mouse hepatocytes, reducing liver damage in mice with acute liver failure and slowing the progression of the illness. In recent years, some scholars have found that AAT can also promote wound healing by reducing the degree of wound inflammation, but it has not been reported that it is associated with lumbar disc herniation. In this study, it was found that human *α*-1 antitrypsin protein (HAAT) was significantly downregulated before and after integrated traditional and western medicine treatment of lumbar disc herniation, indicating that human *α*-1 antitrypsin protein may be involved in the treatment process, but its expression mechanism and regulation are not clear.

## 4. Results

### 4.1. Differentiated Free Radical Metabolism

Fourteen differentially expressed proteins annotated to related signal pathways were screened, and the interaction between proteins was analyzed. It was found that some differentially expressed proteins had broad relationship with other proteins; that is, they played a nodal role in molecular expression. Fibronectin 1, apolipoprotein C3, apolipoprotein A-II, apolipoprotein A-IV, apolipoprotein A-I, apolipoprotein A-II, apolipoprotein A-I, apolipoprotein A-I, apolipoprotein A-I, apolipoprotein B, complement C3, human-1 antitrypsin protein, and c DNA proteins are concentrated in the functional network, and they may play a key role in the biological foundation of combined traditional and western medicine in the treatment of LIDP. The most frequent illness in clinic is lumbar disc herniation (LIDP), which is also the most common disease in spinal orthopaedics. In recent years, with the influence of work and life style, it shows an increasing trend year by year. Young and middle-aged manual workers have a high incidence of lumbar disc herniation, whose main clinical manifestations are lumbar and leg pain, scoliosis, dyskinesia, lower limb pain, and numbness, often occurring repeatedly, bringing a heavy burden to patients. The main cause of lumbar disc herniation is intervertebral disc degeneration caused by changes in the microstructure of intervertebral disc tissue, nucleus pulposus herniation, and then compression or stimulation to related nerves, resulting in a series of pains and dysfunctions, seriously affecting the quality of life of patients. The study found that there was no significant difference in the long-term effect of surgical and nonoperative treatment in patients with lumbar disc herniation.

At present, it is recognized that the main treatment of lumbar disc herniation is nonoperative treatment. On the other hand, proteomics studies the characteristics of proteins from a macroperspective, including protein mediation, response, function, composition, translation, and interaction between proteins. The results comparison between worst and excellent conditions can be seen in Figure 6. This offers information on the incidence, progression, and molecular metabolism of illnesses at the protein level, which may help us comprehend the information of proteins in a certain condition and investigate the connection between proteins and disease occurrence and progression. Therefore, in order to find the comprehensive pathophysiological mechanism of lumbar disc herniation, it is necessary to identify the differentially expressed proteins. Proteomics technology has developed rapidly in recent years, and there has been an opportunity to synchronously screen differentially expressed proteins associated with disease occurrence, diagnosis, and treatment and posttreatment assessment. This technique is based on a high-throughput high-performance liquid chromatography-tandem mass spectrometry (HPLC-MS) approach that can detect the relative or absolute concentration of proteins in up to 8 distinct samples concurrently and with a high protein detection rate. It is especially suitable for the study of low-abundance proteins that determine treatment-related differences. Therefore, the study of proteomics technology in the field of treatment of lumbar disc herniation can provide new ideas for the study of the mechanism of treatment of lumbar disc herniation. This study is based on proteomics to carry out the study of nonoperative treatment of lumbar disc herniation with integrated traditional and western medicine, in order to find the difference of protein expression both before and after treatment and then provide a molecular basis for elucidating the related mechanism of integrated traditional and western medicine treatment of the disease.

### 4.2. Discussion

Fourteen differentially expressed proteins annotated to related signal pathways were screened, and the interaction between proteins was analyzed. It was found that some differentially expressed proteins had broad relationship with other proteins; that is, they played a nodal role in molecular expression. The functional network contains fibronectin 1, apolipoprotein C3, apolipoprotein A-II, apolipoprotein A-IV, apolipoprotein A-I, apolipoprotein B, complement C3, human-1 antitrypsin protein, and DNA proteins, which may play an important role in the biological basis of integrated traditional and western medicine in the treatment of LIDP. The most frequent illness in clinic is lumbar disc herniation (LIDP), which is also the most common disease in spinal orthopaedics. In recent years, with the influence of work and life style, it shows an increasing trend year by year. Young and middle-aged manual workers have a high incidence of lumbar disc herniation, whose main clinical manifestations are lumbar and leg pain, scoliosis, dyskinesia, lower limb pain, and numbness, often occurring repeatedly, bringing a heavy burden to patients. The main cause of lumbar disc herniation is intervertebral disc degeneration caused by changes in the microstructure of intervertebral disc tissue, nucleus pulposus herniation, and then compression or stimulation to related nerves, resulting in a series of pains and dysfunctions, seriously affecting the quality of life as shown in Figure 7. The study found that there was no significant difference in the long-term effect of surgical and nonoperative treatment in patients with lumbar disc herniation.

At present, it is recognized that the main treatment of lumbar disc herniation is nonoperative treatment. On the other hand, proteomics studies the characteristics of proteins from a macroperspective, including protein mediation, response, function, composition, translation, and interaction between proteins. This offers information on the incidence, progression, and molecular metabolism of illnesses at the protein level, which may help us comprehend the information of proteins in a certain condition and investigate the connection between proteins and disease occurrence and progression. Therefore, in order to find the comprehensive pathophysiological mechanism of lumbar disc herniation, it is necessary to identify the differentially expressed proteins. Proteomics technology has developed rapidly in recent years, and there has been an opportunity to synchronously screen differentially expressed proteins associated with disease occurrence, diagnosis, and treatment and posttreatment assessment. This technique is based on a high-throughput high-performance liquid chromatography-tandem mass spectrometry (HPLC-MS) approach that can detect the relative or absolute concentration of proteins in up to 8 distinct samples concurrently and with a high protein detection rate. It is especially suitable for the study of low-abundance proteins that determine treatment-related differences. Therefore, the study of proteomics technology in the field of treatment of lumbar disc herniation can provide new ideas for the study of the mechanism of treatment of lumbar disc herniation. This study is based on proteomics to carry out the study of nonoperative treatment of lumbar disc herniation with integrated traditional and western medicine, in order to find the difference of protein expression both before and after treatment and then provide a molecular basis for elucidating the related mechanism of integrated traditional and western medicine treatment of the disease.

Hemoglobin is an important protein in the components of human red blood cells, which can carry the corresponding oxygen in and out of various tissues and organs in the body. Normal hemoglobin is formed by two groups of globin peptide chain and four heme combination subunits, while the globin peptide chain of human hemoglobin can be divided into six types: *α*, *β*, *γ*, *δ*, *ε*, and *ζ* chain. Structural changes in peptide chains can cause changes or abnormalities in hemoglobin biological activity and related physiological functions, and structural abnormalities can occur in any kind of globin chain. At present, more than 1000 varieties of hemoglobin have been found, covering a variety of globin chains. Most of the variants have genetic characteristics, and only a small number of variants can produce clinical symptoms.

At present, the deletion of *α*-globin gene mainly points to *α*-thalassemia, which is a group of hereditary hemolytic diseases caused by the imbalance of one or more syntheses of globin peptide chain in hemoglobin due to the defect or deletion of globin gene. Despite the fact that no studies have linked the hemoglobin-1 globin chain variant gene mutation to lumbar disc herniation, some researchers performed a cross-sectional control study on the blood routine test indices of 502 lumbar disc herniation patients and 3625 healthy individuals. It was found that the levels of red blood cells and hemoglobin in peripheral blood of patients with lumbar disc herniation decreased significantly. It is suggested that patients with lumbar disc herniation may have chronic red blood cell consumption. The *ß* chain of hemoglobin is mainly composed of more than 100 amino acid residues, in which the first type cysteine is easily oxidized to form mixed disulfides and sulfides, which affects the stability of hemoglobin as shown in Figure 8. Generally speaking, the defect of hemoglobin *ß* chain is mainly *ß*-thalassemia. There is currently no evidence that hemoglobin-globin is linked to lumbar disc herniation, but it was discovered that hemoglobin-globin showed significant differences in pathological changes in patients with ankylosing spondylitis at various stages and in the screening and identification of differentially expressed proteins in serum of patients with ankylosing spondylitis at various stages. In this study, it was found that hemoglobin *α*-1 globin chain variant and hemoglobin *ß* globin were upregulated before and after integrated traditional and western medicine treatment of lumbar disc herniation, suggesting that hemoglobin *α*-1 globin chain variant and hemoglobin *ß* globin may play a role in the physiological and pathological development of LIDP, but its mediation and regulation mechanism is not clear. Further studies are needed to verify whether it may become a potential molecular marker for the treatment of lumbar disc herniation.

## 5. Conclusion

The study of proteomics technology in the field of treatment of lumbar disc herniation can provide new ideas for the study of the mechanism of treatment of lumbar disc herniation. This study is based on proteomics to carry out the study of nonoperative treatment of lumbar disc herniation with integrated traditional and western medicine, in order to find the difference of protein expression both before and after treatment and then provide a molecular basis for elucidating the related mechanism of integrated traditional and western medicine treatment of the disease. Lumbar disc herniation is a common lumbar disease in clinic, which is related to improper use of lumbar vertebrae and osteoporosis. Surgical removal of nucleus pulposus and maintenance of lumbar structural stability are important for the treatment of lumbar disc herniation. At present, in clinical percutaneous intervertebral foramen endoscopic surgery for lumbar disc herniation, interlaminar and intervertebral foramen approaches can be selected. Different approaches have different degrees of difficulty in the treatment of lumbar disc herniation, and the clinical effects that may be obtained are different. Apolipoprotein A-IV, apolipoprotein B, and apolipoprotein Amuri are the proteins involved in this pathway, with apolipoprotein B being the most highly expressed and apolipoprotein A-IV and apolipoprotein Amuri being the least.

## Figures and Tables

**Figure 1:** The detection of lumbar disc herniation.

**Figure 2:** CT mapping for the lumbar disc herniation.

**Figure 3:** The complement and coagulation cascade for the lumbar disc herniation. (a) Arterial occlusion. (b) Arteriosclerosis.

**Figure 4:** The bromine domain protein.

**Figure 5:** The comparison results between observation and experiment results.

**Figure 6:** The results comparison between worst and excellent conditions.

**Figure 7:** Comparison of free radical release processes.

**Figure 8:** The treatment efficiencies for different types.

## Data Availability

The data used to support the findings of this study are included within the article.

## References

[1] Tobert D. G., Antoci V., Patel S. P., Saadat E., Bono C. M. (2017). Adjacent segment disease in the cervical and lumbar spine. *Clinical Spine Surgery: A Spine Publication*.

[2] Murphy M. E., Mccutcheon B. A., Grauberger J. (2018). Allograft versus autograft in cervical and lumbar spinal fusions: an examination of operative time, length of stay, surgical site infection, and blood transfusions. *Journal of Neurosurgical Sciences*.

[3] Jones J. H., Singh N., Nidecker A., Li C.-S., Fishman S. (2017). Assessing the abetween radiologic and clinical measurements of lumbar and cervical epidural depths in patients undergoing prone interlaminar epidural steroid injection. *Anesthesia & Analgesia*.

[4] Huang H., Nightingale R. W., Dang A. B. C. (2018). Biomechanics of coupled motion in the cervical spine during simulated whiplash in patients with pre-existing cervical or lumbar spinal fusion. *Bone & Joint Research*.

[5] Morishita Y., Buser Z., D’Oro A., Shiba K., Wang J. C. (2018). Clinical relationship of degenerative changes between the cervical and lumbar spine. *Asian Spine Journal*.

[6] Vydra D., Hynes A., Clements N. (2019). Current practice trends in image guidance during lumbar and cervical t epidural steroid injections. *Pain Medicine*.

[7] Jabłońska R., Ślusarz R., Królikowska A., Haor B., Antczak A., Szewczyk M. (2017). Depression, social factors, and pain perception before and after surgery for lumbar and cervical degenerative vertebral disc disease. *Journal of Pain Research*.

[8] Goldschmidt E., Angriman F., Ferreyro B. (2018). Design and testing of 2 novel scores that predict global sagittal alignment utilizing cervical or lumbar plain radiographs. *Neurosurgery*.

[9] Epping R., Verhagen A. P., Hoebink E. A., Rooker S., Scholten-Peeters G. G. M. (2017). The diagnostic accuracy and test-retest reliability of the Dutch PainDETECT and the DN4 screening tools for neuropathic pain in patients with suspected cervical or lumbar radiculopathy. *Musculoskeletal Science and Practice*.

[10] Shim E., Lee J. W., Lee E., Ahn J. M., Kang Y., Kang H. S. (2017). Fluoroscopically guided epidural injections of the cervical and lumbar spine. *RadioGraphics*.

[11] Mizutani J., Verma K., Endo K. (2018). Global spinal alignment in cervical kyphotic deformity: the importance of head position and thoracolumbar alignment in the compensatory mechanism. *Neurosurgery*.

[12] Pobloth A.-M., Duda G. N., Giesecke M. T., Dienelt A., Schwabe P. (2017). High-dose recombinant human bone morphogenetic protein-2 impacts histological and biomechanical properties of a cervical spine fusion segment: results from a sheep model. *Journal of Tissue Engineering and Regenerative Medicine*.

[13] Hsu H.-T., Yue C.-T., Teng M.-S. (2019). Immuohistochemical score of matrix metalloproteinase-1 may indicate the severity of symptomatic cervical and lumbar disc degeneration. *The Spine Journal*.

[14] Phan K., Phan P., Stratton A., Kingwell S., Hoda M., Wai E. (2019). Impact of resident involvement on cervical and lumbar spine surgery outcomes. *The Spine Journal*.

[15] Sohn S., Chung C. K., Han I., Park S. B., Kim H. (2018). Increased bone mineral density in cervical or thoracic diffuse idiopathic skeletal hyperostosis (dish): a case-control study. *Journal of Clinical Densitometry*.

[16] Hk V., Dellen V. (2018). A perspective on the use of an enhanced recovery program in open, non-instrumented day surgery for degenerative lumbar and cervical spinal conditions. *Journal of Neurosurgical Sciences*.

[17] Sharpe E. E., Gazelka H. M., Arendt K. W. (2019). Postdural puncture headache with extensive spread of lumbar-cervical epidural cerebrospinal fluid. *Canadian Journal of Anesthesia/Journal canadien d’anesthésie*.

[18] Patel E. A., Perloff M. D. (2018). Radicular pain syndromes: cervical, lumbar, and spinal stenosis. *Seminars in Neurology*.

[19] Joswig H., Neff A., Ruppert C., Hildebrandt G., Stienen M. N. (2018). Repeat epidural steroid injections for radicular pain due to lumbar or cervical disc herniation. *The Bone & Joint Journal*.

[20] Akbar M., Almansour H., Lafage R. (2018). Sagittal alignment of the cervical spine in the setting of adolescent idiopathic scoliosis. *Journal of Neurosurgery: Spine*.

[21] Zhao Y., Talha M. (2021). Evaluation of food safety problems based on the fuzzy comprehensive analysis method. *Food Science and Technology*.

[22] Talha M. (2020). Mediating effects of reflexivity of top management team between team processes and decision performance. *Azerbaijan Journal of Educational Studies*.

[23] Uehara M., Takahashi J., Ikegami S., Kuraishi S., Futatsugi T., Kato H. (2017). Screw perforation rates in 359 consecutive patients receiving computer-guided pedicle screw insertion along the cervical to lumbar spine. *European Spine Journal*.

[24] Ebot J., Nottmeier E. (2019). Tumoral calcinosis of the lumbar and cervical spine. *Journal of Clinical Neuroscience*.

